The article "The Influence of Repeated Drop Jump Training on Countermovement Jump Performance" was published in 2022. Journal: Appl Bionics Biomech.

# The Influence of Repeated Drop Jump Training on Countermovement Jump Performance

**DOI:** 10.1155/2022/9609588

**Published:** 2022-02-21

**Authors:** Lin He, Yu-Ge Li, Chou Wu, Shun Yao, Yu Su, Guo-Dong Ma, I-Lin Wang

**Affiliations:** ^1^Training Science in Physical Education College, Jilin Sport University, Changchun, 130022 Jilin, China; ^2^Graduate Institute, Jilin Sport University, Changchun, 130022 Jilin, China; ^3^Human Movement Science College, Jilin Sport University, Changchun, 130022 Jilin, China; ^4^Health Technology College, Jilin Sport University, Changchun, 130022 Jilin, China

## Abstract

Countermovement jump (CMJ) is used to assess athletic performance of the lower limbs. Drop jump (DJ) is an effect training method that can improve athlete's jumping performance. The main purpose of this study is to explore the effects of different drop jump heights (DJH)30, DJH40, and DJH50 cm for 250 drop jumps (DJs250) on CMJ. Eighteen male athletes were selected as subjects. After the 50th, 100th, 150th, 200th, and 250th DJs, perform 5 groups of CMJ (the average of 3 times for each group) and record them as the 50th, 100th, 150th, 200th, and 250th CMJ jumps (CMJs50, CMJs100, CMJs150, CMJs200, and CMJs250). The BTS motion capture system and two force plates are used to record data. The MATLAB software was used to analyze data through one-way ANOVA repeated measures. If there is a significant difference, the LSD method is used for post hoc comparison. Jump height (JH), contact time (CT), reaction intensity index (RSI), average rate of force development (ARFD), left average rate of force development (LARFD), and right average rate of force development (RARFD) of CMJs50, CMJs100, CMJs150, and CMJs200 at DJH50 were greater than those at DJH40 and DJH30 (all *p* < 0.05). DJH50 height and DJs200 training times can improve SSC mechanism and improve athlete CMJ performance.

## 1. Introduction

Countermovement jumps (CMJs) are coordinated movements often used to evaluate lower extremity jump ability and sports performance [1]. CMJ involves rapid and powerful stretching of the lower extremity muscles immediately after shortening. The continuous concentric contraction and eccentric contraction of the muscles are called the stretch-shortening cycle (SSC) [2]. Past studies have found that using the SSC elastic energy mechanism increases the strength, speed, and muscle activation of the CMJ eccentric phase and increases the jump height during the CMJ concentric phase [3]. Thus, applying the SSC mechanism can enhance the muscle strength of the lower extremities and the jumping height in the CMJ to improve athletic performance. In addition, previous studies have found that drop jumps (DJs) are an effective plyometric training (PT) and SSC training method, currently being widely used to improve jumping ability and leg strength to improve athletic performance [3, 4]. Therefore, DJ training can enhance the SSC mechanism to improve CMJ performance.

The article "The Influence of Repeated Drop Jump Training on Countermovement Jump Performance" was published in 2022. Journal: Appl Bionics Biomech.

Past studies have found that the jump height of DJ training from 50 cm and 60 cm platforms was lower than 20 cm and 30 cm [5]. After 200 DJs at 30 cm, 40 cm, and 50 cm, it was found that the 30 cm jump height could effectively store elastic potential energy by SSC mechanism and improve the jumping performance [2]. Therefore, training at the optimal height can better improve the vertical jumping performance and protect the lower extremities from injury. In addition, 6-week repeat DJ training of 90 drop jumps at drop heights of 50 cm and 100 cm increased the jump height of the CMJ by 4.8 cm and 5.6 cm, respectively [6]. After 7 weeks of repeat DJ training of 60 drop jumps at drop heights of 20 cm, 40 cm, and 60 cm, the 2.4 km endurance running time decreased by 1.9%, and the jump height of the CMJ increased by 4.3% [7]. Thus, 6 or 7 weeks of repeated long-term DJ training at different drop heights and at different times can increase the jump height of CMJs and enhance the endurance performance of athletes. Therefore, repeat DJ training and long-term DJ training can be used as an effective PT training method, which has a positive impact on CMJ performance and muscle endurance development.

DJs can be used to examine changes in mechanical risk factors for potential anterior cruciate ligament (ACL) injury [8]. Previous studies have found that repetitions of 100 countermovement jumps can cause fatigue of the extensor muscles and reduce the jump height of the CMJ by 14% [9]. After repeated DJ training of 200 drop jumps at a drop height of 60 cm within 24 hours and repeated DJ training of 100 drop jumps at a drop height of 35 cm within 48 hours, the jump height of CMJ and the extensor muscle strength of the lower extremity decreased [10]. Repeat DJ training of 100 drop jumps at a drop height of 60 cm decreases muscle function and the jump height of the CMJ [11]. Thus, excessive repetitive DJ training can cause muscle fatigue and increase the risk of lower extremity muscle damage, which affects the performance of CMJs. However, appropriate DJ training can increase the jump height and reduce the risk of injury [8]. Therefore, excessive repetitive DJ training causes muscle fatigue and increases the risk of lower extremity muscle damage, which affects CMJ performance. Appropriate DJ training reduces muscle fatigue and the risk of injury, which improves athletic performance.

Previous studies have found that excessive drop height of the DJ will reduce the muscle activation of the quadriceps and hamstrings, which will increase the risk of injury during the landing phase of the DJ [12]. When the drop height exceeds 60 cm, it may mean the lack of biomechanical efficiency and the potentially increased risk of injury efficiency [5]. Exceeding the optimal drop height will cause knee joint instability and increase the risk of lower extremity injuries [13]. Therefore, excessive drop height will increase the risk of lower extremity injuries and decrease sports performance. However, a lower drop height of the DJ cannot achieve the desired training effect and can cause injury [14]. Past studies have found that after DJ training of 10 drop jumps at a drop height of 75 cm for 5 minutes, the jump height of the CMJ increased by 5.5% [15]. After DJ training of 5 drop jumps at a drop height of 30 cm for 4 minutes, 8 minutes, and 12 minutes, the jump height of the CMJ increased by 2.5 cm, 2.1 cm, and 2.2 cm, respectively [16]. Thus, short-term DJ training at different drop heights can increase the jump height of the CMJ. In addition, a previous study found that after 7 weeks of training at drop heights of 10 cm, 20 cm, 30 cm, 40 cm, and 50 cm, the jump height of the CMJ increased by 16.7% for young football players [17]. During DJ training of 50 drop jumps at drop heights of 35 cm and 50 cm, the jump height of the CMJ increased by 13.2% [18]. Thus, long-term DJ training has effectively improved the performance of the CMJ. Therefore, both short-term and long-term DJ trainings at an appropriate drop height can improve CMJ performance. DJ training at an inappropriate drop height will induce lower extremity injuries and impair the jump height of the CMJ.

The article "The Influence of Repeated Drop Jump Training on Countermovement Jump Performance" was published in 2022. Journal: Appl Bionics Biomech.

DJ training at appropriate drop height can increase the jump height of the CMJ by the SSC mechanism, which would prevent lower extremity injuries and enhance muscle endurance to improve athletic performance. Therefore, the main purpose of this study was to explore the jump performance of CMJs after repeat DJ training at different heights. This experiment hypothesized that the athletic performance of the CMJ increases with the drop height of the DJ.

## 2. Methods

### 2.1. Subjects

Eighteen male athletes (age: 20.66 ± 1.37 years old; height: 1.75 ± 0.05 m; weight: 79.79 ± 12.30 kg) from Jilin Sport University were included as subjects. None of the subjects had a lower extremity injury that affected their jumping ability within the past 6 months. The patients were encouraged not to perform physical exercise for at least 48 hours before the test. The subjects were informed of the benefits and all of the procedures and risks of the study and signed the consent form. This study was approved by the regional ethics committee (JLSU-IRB2020005).

The article "The Influence of Repeated Drop Jump Training on Countermovement Jump Performance" was published in 2022. Journal: Appl Bionics Biomech.

### 2.2. Procedures

All subjects needed to be familiar with the experimental procedures and jumping skills in advance. In this experiment, the three drop jump heights (DJH)30 cm, DJH40 cm, and DJH50 cm were separated by 7 days and randomly chosen. The subjects wore the same experimental running shoes and warmed up on a treadmill at a speed of 8 km/h for 5 minutes. After warming up, all subjects completed a set of drop jumps (50 DJs in each set) followed by a set of countermovement jumps (3 CMJs in each set). All subjects need to perform 5 sets of DJs (250 total) and 5 sets of CMJs (15 total). After performing 50 DJs, subjects performed a set of CMJs which was recorded as CMJs50. After performing a set of CMJs, subjects performed 50 DJs again. Then, subjects performed a set of CMJs which was recorded as CMJs100. Subsequently, CMJs were recorded as CMJs150, CMJs200, and CMJs250. CMJs50, CMJs100, CMJs150, CMJs200, and CMJs250 were used for data analysis. Each DJ and CMJ were performed after resting for 10 seconds and 1 minute. During CMJ, the subjects should stand on the two force plates to maintain a stable upright posture, then quickly squat, swing their arms up, and jump upward with maximum effort. Both of their feet should naturally land on the ground and fall on the two force plates as symmetrically as possible. During DJ, the subjects stand on a fixed high platform with their hands on their hips; they leave the platform with the dominant leg and land on the two force plates after their feet naturally descend and then at their maximum speed and strength jump and fall. The specific process is shown in Figure 1 below.

### 2.3. Data Collection

Ten infrared motion capture cameras (SMART-DX400, BTS, Milano, Italy) were used to collect the kinematic data at a sampling frequency of 200 Hz. Two force-measuring plates (BTS P6000, BTS Bioengineering, Italy) installed on the ground at 40 cm × 60 cm collected dynamic data at a sampling frequency of 400 Hz. The subjects used 19 (19 mm diameters) reflective balls from the Helen Hayes lower limb model to mark the 7-segment rigid link model of the lower extremity [19].

### 2.4. Data Analysis

Markers were located on the anterior superior iliac spine, sacrum, thigh, femoral lateral epicondyle center, tibia, lateral medial malleolus, second metatarsal, and heel. Each joint segment (pelvis, knee, ankle, and foot) was defined to form a kinematic model [20]. The kinematic data were low-pass filtered using a fourth-order Butterworth filter with a cutoff frequency of 12 Hz, and the kinetic data were low-pass filtered using a fourth-order Butterworth filter with a cutoff frequency of 50 Hz [21]. The measurement parameters include jump height (JH), contact time (CT), relative strength index (RSI), average force rate (ARFD), left average force rate (LARFD), and right average force rate (RARFD),JH = *gT*^2^/8(*g* = 9.81 ms^−2^). CT was defined as the time from initial ground contact to toe-off during the foot ground contact phase. RSI is the ratio of JH to CT. ARFD is the value subtracted 1 from the ratio of the maximum vGRF−body weight to time of maximum vGRF−time at which force reach the body weight during push-off phase [22].

The article "The Influence of Repeated Drop Jump Training on Countermovement Jump Performance" was published in 2022. Journal: Appl Bionics Biomech.

### 2.5. Statistical Analysis

All data are expressed as the mean ± standard deviation. MATLAB (R2019A; Math Works, Inc., Natick, MA) software was used to analyze the data. One-way repeated-measures ANOVA was used for the data analysis of the CMJs (CMJs50, CMJs100, CMJs150, CMJs200, and CMJs250). When the results are significant, the LSD is used to perform post hoc tests to compare different drop heights (DJH30, DJH40, and DJH50). *p* < 0.05 indicates significance. The effect size (ES) was used to determine whether the difference was actually a clinically relevant difference. The modified Cohen scale was used to determine the variation of the three heights: 0.2 represents a negligible difference, 0.2-0.6 represents a small difference, 0.6-1.2 represents a medium difference, and 1.2-2.0 represents a large difference [23].

## 3. Results

The experimental results showed that the JH, CT, RSI, ARFD, LARFD, and RARFD of CMJs50, CMJs100, CMJs150, and CMJs200 at DJH50 were greater than those at DJH30 and DJH40. The JH, CT, RSI, ARFD, LARFD, and RARFD of CMJs250 at DJH50 were smaller than those at DJH30 and DJH40.

The experimental results showed that (Figure 2) the JH, CT, RSI ARFD, LARFD, and RARFD of CMJs50, CMJs100, CMJs150, CMJs200, and CMJs250 were significantly different among the three different drop heights (*p* < 0.05).

The postmortem comparison showed that the JH of CMJs50, CMJs100, CMJs150, and CMJs200 at DJH50 was greater than that at DJH40 and DJH30 (all *p* < 0.001; ES = 0.90 − 1.00). But the JH for CMJs250 at DJH50 was smaller than that at DJH40 and DJH30 (*p* = 0.040; ES = 0.20 − 0.70) (Figure 2(a)). The postmortem comparison showed that the CT values of CMJs50, CMJs100, CMJs150, and CMJs200 at DJH50 were greater than those at DJH40 and DJH30 (all *p* < 0.001; ES = 0.60 − 1.35). The CT of CMJs250 at DJH50 was smaller than that at DJH30 and DJH40 (*p* = 0.014; ES = 0.40 − 0.55) (Figure 2(b)). The postmortem comparison showed that the RSIs of CMJs50, CMJs100, CMJs150, and CMJs200 at DJH50 were greater than those at DJH40 and DJH30 (all *p* < 0.001; ES = 0.60 − 1.25). The RSI of CMJs250 at DJH50 was smaller than that at DJH30 and DJH40 (*p* = 0.037; ES = 0.40 − 0.65) (Figure 2(c)).

The article "The Influence of Repeated Drop Jump Training on Countermovement Jump Performance" was published in 2022. Journal: Appl Bionics Biomech.

The postmortem comparison showed that the ARFD of CMJs50, CMJs100, CMJs150, and CMJs200 at DJH50 was greater than that at DJH40 and DJH30 (all *p* < 0.04; ES = 0.10 − 1.2) (Figure 2). The ARFD of CMJs250 at DJH50 was smaller than that at DJH40 and DJH30 (*p* < 0.001; ES = 0.50 − 1.10) (Figure 2(d)). The post hoc comparison showed that the LARFD of CMJs50, CMJs100, CMJs150, and CMJsDJ200 at DJH50 was greater than that at DJH40 and DJH30 (all *p* < 0.04; ES = 0.20 − 1.40). The LARFD of CMJs250 at DJH50 was smaller than that at DJH40 and DJH30 (*p* = 0.002; ES = 0.30 − 0.85) (Figure 2(e)). The postmortem comparisons showed that the RARFDs of CMJs50, CMJs100, CMJs150, CMJs150, and CMJ200DJ at DJH50 were greater than those at DJH40 and DJH30 (all *p* < 0.05; ES = 0.07 − 1.00). The RARFD of CMJs250 at DJH50 was smaller than that of DJH40 and DJH30 (*p* < 0.001; ES = 0.60 − 1.00) (Figure 2(f)).

## 4. Discussion

The purpose of this study was to compare the effects of repeated DJ training at different drop heights (DJH30, DJH40, and DJH50) on CMJ performance. The main finding of this study is that the JH, CT, RSI, LARFD, RARFD, and ARFD of CMJs50, CMJs100, CMJs150, CMJs150, and CMJ200DJ at DJH50 are all greater than those at DJH40 and DJH30. JH, CT, RSI, LARFD, RARFD, and ARFD of CMJs250 are smaller than those at DJH40 and DJH30. The DJs200 training at DJH50 can effectively use the SSC mechanism to improve CMJ performance. DJs250 training at DJH50 can cause muscle fatigue and reduce CMJ performance.

This study found that the JH of CMJs50, CMJs100, CMJs150, and CMJs200 at DJH50 was greater than that at DJH40 and DJH30. Previous studies have found that the jump heights of DJH40 and DJH60 are greater than those of DJH20, and different drop heights may increase jumping performance and neuromuscular adaptations [24]. The jump height at DJH60 was greater than that at DJH20 and DJH40, and DJH60 could increase the muscle stretch load and muscle elastic potential energy to increase the jump height [25]. Therefore, DJ training from an appropriate drop height may enhance the SSC mechanism and stretch load to increase athletic performance. In this study, within the DJs200, training at DJH50 increased the stretch load and neuromuscular adaptability to improve the JH of CMJs50, CMJs100, CMJs150, and CMJs200. In addition, the JH of CMJs250 at DJH50 is smaller than that at DJH40 and DJH30. Repeat DJs200 from a drop height of 60 cm causes muscle fatigue and decreases the JH of the CMJ [10]. Excessive DJs200 from a drop height of 20 cm causes muscle fatigue to decrease the JH of the CMJ [26]. Therefore, excessive DJs200 may cause muscle fatigue and decrease the JH of CMJs. In this study, DJs250 training at DJH50 caused muscle fatigue and decreased the JH of CMJs250. Therefore, within the DJs200, training at DJH50 increases the stretch load and neuromuscular adaptability to improve the JH of CMJs. DJs250 training at DJH50 caused muscle fatigue and decreased the JH of the CMJs.

The article "The Influence of Repeated Drop Jump Training on Countermovement Jump Performance" was published in 2022. Journal: Appl Bionics Biomech.

This study found that the CT of CMJs50, CMJs100, CMJs150, and CMJs200 at DJH50 was greater than that at DJH40 and DJH30. Previous studies have found that the CT at a drop height of 60 cm is greater than that of 5 cm, 30 cm, and 45 cm, and a 60 cm drop height increases the absorption of the impact force by a longer CT [27]. The CT at a drop height of 40 cm is greater than that of 60 cm and 20 cm, and the 40 cm drop height increases the knee power due to a longer CT [28]. Therefore, DJ training may increase the absorbed impact force and knee power by promoting a longer CT. In this study, within DJs200, training at DJH50 increased the absorption of the impact force and knee power by increasing the CT of CMJs50, CMJs100, CMJs150, and CMJs200 at DJH50. In addition, the CT of CMJs250 at DJH50 was smaller than that at DJH40 and DJH30. Previous studies have found that repeat DJs100 from a drop height of 40 cm causes muscle fatigue to decrease the CT [29]. Therefore, in this study, DJ250 training at DJH50 caused muscle fatigue and decreased the CT of CMJ250 at DJH50. Therefore, within the DJs200 training at DJH50, the absorption of the impact force is increased to improve the CT of the CMJ. DJs250 training at DJH50 caused muscle fatigue and decreased the CT of the CMJ.

This study found that the RSI of CMJs50, CMJs100, CMJs150, and CMJs200 at DJH50 was greater than that at DJH40 and DJH30. RSI is an index used to evaluate training effects, and it is related to JH and CT. It increases with increasing JH and decreasing CT. Previous studies have found that a drop height in the range of 20 cm to 50 cm can increase the RSI [30]. Appropriate drop heights can increase the efficiency of the SSC and the jump height of the DJ, thereby increasing the RSI [27]. In this study, within DJs200, training at DJH50 increased the exercise efficiency of the SSC and jump height of the CMJ, which increased the RSI of CMJs50, CMJs100, CMJs150, and CMJs200. However, the RSI of CMJs250 at DJH50 is smaller than that at DJH40 and DJH30. Previous studies have found that the JH of CMJ decreased after DJs200, and high-intensity load and repetitive DJ training led to muscle damage [10]. Muscle fatigue caused by excessive DJ training decreases the RSI of the CMJ. In this study, DJs250 training at DJH50 may cause muscle fatigue and reduce the RSI of CMJs250. Therefore, within DJs200, training at DJH50 increases the efficiency of the SSC and jump height of the CMJ, which increases the RSI of the CMJ. DJ250 training at DJH50 causes muscle fatigue and reduces the RSI of CMJs250.

The article "The Influence of Repeated Drop Jump Training on Countermovement Jump Performance" was published in 2022. Journal: Appl Bionics Biomech.

This study found that the ARFD, LARFD, and RARFD of CMJs50, CMJs100, CMJs150, and CMJs200 at DJH50 were greater than those at DJH40 and DJH30. Previous studies have found that the ARFD at DJH60 is greater than that at DJH40 and DJH20, and the drop height of DJH60 can increase the muscle load and elastic potential energy [31]. The RFD of DJH50 is greater than that of DJH35 and DJH20, and the drop height of DJH50 increases the elastic potential energy of muscle and neuromuscular activation to increase RFD [32]. Therefore, DJ training on an appropriate platform can increase the muscle load and elastic potential energy, which will increase the ARFD. In addition, ARFD can determine changes throughout the eccentric phase of CMJs, reflecting the ability of neuromuscular units to stretch quickly before reaching peak GRF [33]. In this study, within DJs200, training at DJH50 increased the muscle load and elastic potential energy, which increased the ARFD, LARFD, and RARFD of CMJs50, CMJs100, CMJs150, and CMJs200 at DJH50. However, this study found that the ARFD, LARFD, and RARFD of CMJs250 at DJH50 were smaller than those at DJH40 and DJH30. Previous studies have found that the RFD of the DJH50 is lower than no load at 30% BM load, and the large external load causes muscle fatigue to decrease the RFD [32]. Therefore, excessive DJ training causes fatigue and reduces ARFD. In this study, DJs250 training at DJH50 caused muscle fatigue and reduced the ARFD, LARFD, and RARFD of CMJs250 at DJH50. Therefore, within DJs200, training at DJH50 increases the muscle load and elastic potential energy, which increases the ARFD, LARFD, and RARFD of CMJ. DJs250 training at DJH50 caused muscle fatigue and reduced the ARFD, LARFD, and RARFD of CMJs.

### 4.1. Limitations

The limitation of this study may be that the subjects were all athletes, and their sports performance may be better than in the general population. Therefore, caution should be exercised when extending these findings to different populations. Another limitation may be that this study did not test physiological indicators such as blood lactic acid. Future research will focus on these aspects.

## 5. Conclusion

In summary, the JH, CT, RSI, LARFD, RARFD, and ARFD of CMJs50, CMJs100, CMJs150, and CMJs200 at DJH50 were larger than those at DJH40 and DJH30. The JH, CT, RSI, LARFD, RARFD, and ARFD of CMJs250 at DJH50 were smaller than those at DJH40 and DJH30. Within DJ200, training at DJH50 increases CMJ performance. DJs250 training at DJH50 causes muscle fatigue to decrease CMJ performance. Therefore, DJs200 training at DJH50 is recommended to prevent muscle fatigue, reduce injury risk, and increase the SSC mechanism and CMJ performance.

The article "The Influence of Repeated Drop Jump Training on Countermovement Jump Performance" was published in 2022. Journal: Appl Bionics Biomech.

## Figures and Tables

**Figure 1:** Schematic diagram of experiment. DJ: drop jump; CMJ: countermovement jump; DJH30: drop jump from 30 cm drop heights; DJH40: drop jump from 40 cm drop heights; DJH50: drop jump from 50 cm drop heights.

**Figure 2:** (a–f) Represent the JH, CT, RSI, ARFD, LARFD, and RARFD during countermovement jumps from three heights at CMJs50, CMJs100, CMJs150, CMJs200, and CMJs250. CMJ: countermovement jump; JH: jump height; CT: contact time; RSI: reactive strength index; ARFD: both feet average rate of force development; LARFD: left foot average rate of force development; RARFD: right foot average rate of force development; DJH30: drop jump from 30 cm drop heights; DJH40: drop jump from 40 cm drop heights; DJH50: drop jump from 50 cm drop heights. † indicates a significant difference from DJH30; ‡ indicates a significant difference from DJH40; § indicates a significant difference from DJH50 (*p* < 0.05).

## Data Availability

The data results are included in the manuscript.

## Abbreviations

DJ: Drop jump
CMJ: Countermovement jump
JH: Jumping height
CT: Contact time
SSC: Stretch-shortening cycle
RSI: Reaction strength index
ARFD: Average rate of force development
LARFD: Left average rate of force development
RARFD: Right average rate of force development.
